This article has been retracted.

# The Efficacy of Needle-Warming Moxibustion Combined with Hyperbaric Oxygen Therapy for Ischemic Stroke and Its Effect on Neurological Function

**DOI:** 10.1155/2022/2204981

**Published:** 2022-02-21

**Authors:** Yonggang Zhu, Xiuhua Zhu, Zhitian Chen, Xueli Cao, Lu Wang, Lin Zang, Weiwei Cao, Tian Sun, Xinyu Bai

**Affiliations:** ^1^Neurorehabilitation Department, The Affiliated Lianyungang Hospital of Xuzhou Medical University, The First People's Hospital of Lianyungang, The First Affiliated Hospital of Kangda College of Nanjing Medical University, Lianyungang Clinical College of Nanjing Medical University, Lianyungang, 222002 Jiangsu Province, China; ^2^Acupuncture and Massage Department, The Affiliated Lianyungang Hospital of Xuzhou Medical University, The First People's Hospital of Lianyungang, The First Affiliated Hospital of Kangda College of Nanjing Medical University, Lianyungang Clinical College of Nanjing Medical University, Lianyungang, 222002 Jiangsu Province, China

## Abstract

**Objective:**

To elucidate the therapeutic efficacy of needle-warming moxibustion (NWM) combined with hyperbaric oxygen therapy (HBOT) in the treatment of patients with ischemic stroke and its effect on neurological function.

**Methods:**

One hundred patients with ischemic stroke admitted to the Xuzhou Medical University Affiliated Hospital of Lianyungang from January 2019 to July 2021 were enrolled. Among them, 45 patients treated with NWM were set as the control group, and the rest 55 patients treated by NWM combined with HBOT were included in the research group. The curative effect, neurological deficit score, activity of daily living (ADL), balance ability, and the levels of serum proinflammatory factors in both groups were observed and recorded. Of them, the neurological deficit of patients was evaluated by the National Institutes of Health Stroke Scale (NHISS), the ADL ability was determined by the Barthel index score, and the balance ability was assessed by the Berg balance scale.

**Results:**

The total effective rate of the research group was higher than that of the control group. Better ADL and balance ability and milder neurologic impairment were determined in the research group compared with the control group. After treatment, the secretion levels of proinflammatory factors such as C-reactive protein (CRP), tumor necrosis factor-*α* (TNF-*α*), and interleukin-8 (IL-8) in the serum of patients in the research group were statistically lower than those before treatment and the control group.

**Conclusions:**

NWM combined with HBOT is effective in the treatment of patients with ischemic stroke, which can not only improve patients' neurological function, ADL, and balance ability but also inhibit serum inflammatory reactions.

## 1. Introduction

Ischemic stroke is an ischemic and hypoxic disabling disease, which accounts for 80% of the total stroke cases with a predilection for males [1, 2]. Its pathology is related to cerebral artery occlusion, which will reduce the cerebral blood flow and cause rapid loss of neurological function, as well as acute hypoxia in the case of blood-brain barrier damage [3]. The pathogenic factors of the disease include age, hypertension, diabetes, and family history of cerebrovascular diseases. [4, 5]. According to epidemiological statistics, the prognosis of ischemic stroke is not ideal, with 27% of vascular events occurring within 1 year and 45% within 5 years [6]. Currently, there is no effective treatment for ischemic stroke, and the conventional treatment schemes include anticoagulation, neuroprotective drugs, and platelet anticoagulation drugs [7–9]. However, the above treatments have disadvantages such as long cycle and slow onset, with barely satisfactory treatment efficacy [10]. Therefore, this study mainly compares and analyzes the treatment schemes of ischemic stroke, aiming at providing new clinical evidence for the effective containment of the disease.

The acupuncture and moxibustion are important techniques of traditional Chinese medicine, which is simple, effective, and convenient, and can quickly relieve the pain of patients [11]. The needle-warming moxibustion (NWM) is a kind of acupuncture technique, in which the moxa roll is inserted into the needle handle and ignited, so that it can transmit heat to the acupuncture points. It can dredge the meridians, and regulate the blood circulation, with a beneficial effect on the repair of the immune system and the improvement of ischemic diseases [12, 13]. At present, this acupuncture technique has been widely used in the treatment of diseases, such as obstructive pulmonary disease, ankylosing spondylitis, and acute lumbago, and has been confirmed to be effective and safe to curb the clinical symptoms and progression of these diseases [14–16]. Hyperbaric oxygen therapy (HBOT), a therapeutic technique combining high pressure and high oxygen content, can induce neuroplasticity and improve damaged nerve fibers and has been shown to improve the neurocognitive function of patients with chronic stroke [17]. In addition, it can be used for the treatment of patients with the severe craniocerebral injury, which can improve their cognitive function and prognosis by facilitating neurological recovery [18]. At present, there are few clinical studies on the combination therapy of NWM and HBOT in the treatment of patients with ischemic stroke. Accordingly, this study mainly compares and analyzes the therapeutic effects of NWM alone and its combination with HBOT in ischemic stroke and their impacts on patients' neurological function, hoping to provide new strategies for the treatment of the disease.

## 2. Materials and Methods

### 2.1. General Data

A total of 100 patients with ischemic stroke admitted to the Xuzhou Medical University Affiliated Hospital of Lianyungang from January 2019 to July 2021 were selected as the study participants. Of them, 45 patients were treated with NWM and set as the control group, including 30 males and 15 females, with an average age of (61.18 ± 8.31) years. The rest 55 cases were treated with NWM combined with HBOT and set as the research group (the research group), including 40 males and 15 females, with a mean age of (63.12 ± 9.74) years. This study was approved by the Ethics Committee of Xuzhou Medical University Affiliated Hospital of Lianyungang, and all participants knew the purpose of this research and provided informed consent. Inclusion criteria: diagnosis of ischemic stroke; patients with first onset and onset time within 24 hours; treatment-naive patients; patients with tolerance to the treatment; and patients with stable vitals and clear consciousness. Exclusion criteria: those with a family history; those with ischemic attack diseases; those with acute or unstable conditions; pregnant or lactation patients; those with disabilities before onset; those with severe liver and kidney dysfunction; and those with a history of mental illness or mental retardation.

### 2.2. Treatment Methods

#### 2.2.1. NWM

Acupoints Baihui, Fengchi (bilateral), Hoku, Jianshu, Quchi, Shousanli, Chize, Zhongzhu, Houxi, Wangu, Taichong, Zusanli, Sanyinjiao, Juegu, Liangqiu, Fengshi, Xuehai, Qihai ,and Juxu (upper and lower) were selected, among which Hoku, Shousanli, Quchi, Jianyu, Liangqiu, Zusanli, and Juxu (upper and lower) were dotted. Each acupoint was disinfected with 75% ethanol before the acupoint selection. The needle was inserted into the needle handle of a 1.5 cm moxa roll, and then the moxa roll was lit until it burned-out. The NWM treatment at each acupoint lasted for 30 min and was performed once daily. Patients were treated for three four-week courses spaced 5 days apart.

#### 2.2.2. HBOT

The oxygen in the hyperbaric oxygen chamber was set at 0.2 mpa, and the treatment was performed once a day for 80 min each time. The treatment lasted for 3 courses, with a course lasting for 12 days and an interval of 2 days between courses. During the treatment, extra attention was paid to the patient's blood pressure, heart rate, and respiratory status.

### 2.3. Outcome Measures

#### 2.3.1. Efficacy

If the patient is conscious and speaks clearly, with normal mobility and the ability to take care of himself/herself, it is regarded as cured. If the patient is conscious, with ordinary language expression and the ability to take care of himself/herself in a simple life, it is regarded as markedly effective. Effective is defined as the patient is conscious, occasionally absent-minded and inarticulate, and needs assistance in normal life. Ineffective is indicated if the patient is unconscious, with no significant improvement in clinical symptoms and signs from those before treatment. The total effective rate of treatment was the percentage of cured, markedly effective, and effective cases to the total cases.

#### 2.3.2. Neurological Deficit Score

The neurological deficit of patients was evaluated by the National Institutes of Health Stroke Scale (NHISS) [19] before and 4 weeks after treatment. On a 0–42 scale, the score is directly proportional to the degree of neurological impairment.

#### 2.3.3. ADL and Balance Ability

Before and 4 weeks after treatment, the ADL and balance ability of patients were evaluated using the Barthel index score and the Berg Balance Scale, respectively [20]. The Barthel index score ranges from 0 to 100, and the score is proportional to the ADL of patients. The Berg balance scale score ranges from 0 to 56, and higher scores suggest better balance ability.

#### 2.3.4. Serum Proinflammatory Factors

Fasting cubital venous blood was drawn from patients in the early morning before and 4 weeks after treatment to detect the serum proinflammatory factors such as C-reactive protein (CRP), tumor necrosis factor-*α* (TNF-*α*), and interleukin-8 (IL-8) by enzyme-linked immunosorbent assay (ELISA) [21] with the corresponding human ELISA kits (Beijing Biowalls Technology Co., Ltd., Beijing, China, Cat. Nos.: EK-H10077, EK-H12145, EK-H10356). The operation process strictly followed the kit instructions.

### 2.4. Statistical Analysis

The SPSS 22.0 (Bioeasy (Beijing) Technology Co., Ltd., Beijing, China) and GraphPad Prism 6 (Shanghai Universal Biotech Co., Ltd., Shanghai, China) were used for data analysis and image rendering, respectively. Count data, such as gender and age, were recorded in the form of number of cases/percentage (*n*/%) and compared by the chi-square test between groups. Measurement data, such as average age and NHIS score, were expressed as mean ± SD, and the methods for intragroup comparison before and after treatment as well as intergroup comparison were paired *t*-test and independent samples *t*-test, respectively. When *P* < 0.05, the difference was statistically significant.

## 3. Results

### 3.1. There Was no Significant Difference in General Data between the Two Groups

There were no significant differences in general data such as gender, age, average age, hypertension, diabetes, hyperlipidemia, drinking history, smoking history, and marital status between the research group and the control group (*P* > 0.05) (Table 1).

### 3.2. The Therapeutic Effect of Patients Was Significantly Improved after Treatment with NWM Combined with HBOT

In the research group, the number of cases with markedly effective, effective, and ineffective treatment was 20, 15, 17, and 3, respectively, while in the control group, the corresponding number of cases was 12, 15, 6, and 12. The total effective rate was 94.55% in the research group and 73.33% in the control group, with a significant difference between the two groups (*P* < 0.05) (Table 2).

### 3.3. The Neurological Deficit Score of Patients Decreased Significantly after Treatment with NWM Combined with HBOT

We evaluated the degree of neurological deficit of patients in both groups using the NHISS scoring system. The results showed that there was no significant difference in the NHISS score between the two groups before treatment (*P* < 0.05); However, the score was significantly reduced in both groups after treatment and was lower in the research group compared with the control group (*P* < 0.05) (Figure 1).

### 3.4. The ADL and Balance Ability of Patients Enhanced Significantly after Treatment with NWM Combined with HBOT

We evaluated the DLA and balance ability of patients using the Barthel index and the Berg balance scale, respectively. The data showed no statistical difference in Barthel index score and Berg balance scale score before treatment between the two groups (*P* > 0.05), while significantly increased scores of both scales in the two groups after treatment, with higher scores in the research group compared with the control group (*P* < 0.05) (Figure 2).

### 3.5. The Serum Levels of Proinflammatory Factors Reduced Significantly in Patients Treated with NWM Combined with HBOT

We detected and analyzed serum levels of proinflammatory factors such as CRP, TNF-*α*, and IL-8 in both groups of patients. The three serum proinflammatory factors, which showed no significant differences between groups before treatment (*P* < 0.05), reduced significantly in both groups after treatment, with lower parameters in the research group compared with the control group (*P* < 0.05). (Figure 3).

## 4. Discussion

As a common central nervous system disease, the ischemic stroke is one of the major causes of death and disability worldwide [22]. Reportedly, this disease threatens the lives of nearly 4.4 million people every year, and brings an average of $590,000 to $2.3 million in medical expenses to each patient, seriously affecting the quality of life of patients and their families [23]. This study, by analyzing the treatment scheme of ischemic stroke, is of great significance for reducing mortality and optimizing the medical management of these patients.

The NWM, a traditional Chinese medicine therapy that combines acupuncture and moxibustion, can not only activate qi and collaterals but also promote blood circulation and remove stasis, which is feasible for the treatment of diseases caused by qi deficiency and blood stasis such as ischemic stroke [24, 25]. The mechanism of action lies in that NWM can repair the internal environment of the body and promote nerve function recovery by the means of heat conduction via regulating the excitatory and inhibitory signals from central and peripheral nerves [26, 27]. The main acupoints selected are Baihui, Qihai, Zusanli, among which Baihui can balance the imbalance of qi and blood in the brain; Qihai can warm channels and dredge collaterals as well as benefit qi and blood, and Zusanli can promote the blood circulation of lower limbs [28]. Therefore, the three acupoints are of great benefit for regulating the lesion site of patients with ischemic stroke, smoothing qi and blood stasis, and relieving the pain of shoulder and wrist [29]. HBOT, on the other hand, can improve the oxygen diffusion rate by increasing the oxygen content and blood oxygen partial pressure in patients' blood and promote the brain tissue to get rid of anoxia, thus repairing the brain function [30]. The data obtained in this research identified a statistically higher total effective rate in the research group compared with the control group (94.55% VS 73.33%), suggesting that NWM combined with HBOT was more effective than NWM alone in the treatment of ischemic stroke. This may be related to the application of the combination therapy, which not only improves the blood circulation of patients by acupuncture but also restrains the brain cell necrosis related to cerebral hypoxia by HBOT, so the curative effect is more remarkable than that of simple NWM. Second, the combination therapy can significantly improve not only the neurological function but also the ADL and balance ability of patients. The research has shown that NWM can also effectively facilitate the rehabilitation of musculoskeletal tissues, with a significant effect on reducing muscle tension and disability rate of patients [26]. Moreover, we evaluated the effects of the two treatment methods on patients' neuroinflammatory reaction. Evidence has shown that the pathogenesis of ischemic stroke is related to neuroinflammation in the body, and proinflammatory markers, such as CRP, TNF-*α*, and IL-8, can promote the neuroinflammatory response of patients with ischemic stroke, thus aggravating the disease progression [31]. In this study, it was found that NWM combined with HBO intervention had a more prominent effect on CRP, TNF-*α*, IL-8, and other proinflammatory factors. Qing et al. [32] showed in their study that NWM can effectively downregulate the secretion levels of serum-related inflammatory factors, which is similar to our research results.

The novelty of this study lies in confirming that NWM combined with HBOT is effective in treating patients with ischemic stroke, which can significantly improve their neurological function, ADL and balance ability, and inhibit neuroinflammation. However, this study still has some limitations. First, this study lacks the related clinical follow up of the long-term efficacy of patients and the analysis of the patient prognosis, which requires further evaluation. Second, the participants enrolled in this study are mainly Chinese, which may limit the extrapolation of different groups to some extent. Third, this is a small sample retrospective study, and the heterogeneity of patients' conditions may have some influence on the research results. These limitations of this study should be addressed in future studies to further validate our conclusions.

## 5. Conclusion

All in all, while effectively inhibiting neuroinflammation, NWM combined with HBOT is significantly beneficial to the neurological function, ADL and balance ability of patients with ischemic stroke, with a better therapeutic effect than NWM alone, which provides a new choice and basis for the treatment of ischemic stroke.

## Figures and Tables

**Figure 1:** The neurological deficit score of patients decreased significantly after treatment with needle-warming moxibustion combined with hyperbaric oxygen therapy. ^∗∗^ indicates *P* < 0.01.

**Figure 2:** The activity of daily living and balance ability of patients enhanced significantly after treatment with needle-warming moxibustion combined with hyperbaric oxygen therapy. (a) The Barthel index score of patients treated with needle-warming moxibustion combined with hyperbaric oxygen therapy was significantly higher than that before treatment and those treated with needle-warming moxibustion alone. (b) The Berg balance scale score of patients after NWM combined with hyperbaric oxygen therapy was significantly higher than that before treatment and those treated with NWM alone. ^∗∗^ indicates *P* < 0.01.

**Figure 3:** The serum levels of proinflammatory factors reduced significantly in patients treated with needle-warming moxibustion combined with hyperbaric oxygen therapy. (a) The level of CRP in patients treated with needle-warming moxibustion combined with hyperbaric oxygen therapy was significantly lower than that before treatment and those treated with needle-warming moxibustion alone. (b) The level of TNF-*α* in patients treated with needle-warming moxibustion combined with hyperbaric oxygen therapy was significantly lower than that before treatment and those treated with needle-warming moxibustion alone. (c) The level of IL-8 in patients treated with needle-warming moxibustion combined with hyperbaric oxygen therapy was significantly lower than that before treatment and those treated with needle-warming moxibustion alone.^∗∗^ indicates *P* < 0.01.

**Table 1:** Baseline data of patients in the two groups [*n* (%), mean ± SD].

Variables	*n*	Control group (*n* =45)	Research group (*n* =55)	*χ* ^2^/t	*P*
Gender				0.433	0.511
Male	70	30 (66.67)	40 (72.73)		
Female	30	15 (33.33)	15 (27.27)		
Age (years)				0.236	0.627
<60	44	21 (46.67)	23 (41.82)		
≥60	56	24 (53.33)	32 (58.18)		
Average age (years)	100	61.18 ± 8.31	63.12 ± 9.74	1.058	0.293
Hypertension				0.271	0.603
No	73	34 (75.56)	39 (70.91)		
Yes	27	11 (24.44)	16 (29.09)		
Diabetes mellitus				1.207	0.272
No	82	39 (86.67)	43 (78.18)		
Yes	18	6 (13.33)	12 (21.82)		
Hyperlipoidemia				0.258	0.611
No	87	40 (88.89)	47 (85.45)		
Yes	13	5 (11.11)	8 (14.55)		
History of drinking				0.948	0.330
No	73	35 (77.78)	38 (69.09)		
Yes	27	10 (22.22)	17 (30.91)		
History of smoking				1.038	0.308
No	78	33 (73.33)	45 (81.82)		
Yes	22	12 (26.67)	10 (18.18)		
Marital status				0.625	0.429
Single	33	13 (28.89)	20 (36.36)		
Married	67	32 (71.11)	35 (63.64)		

**Table 2:** Efficacy of the two groups [*n* (%)].

Groups	*n*	Cured	Markedly effective	Effective	Ineffective	Total effective rate (%)
Control group	45	12 (26.67)	15 (33.33)	6 (13.33)	12 (26.67)	33 (73.33)
Research group	55	20 (36.36)	15 (27.27)	17 (30.92)	3 (5.45)	52 (94.55)
*χ* ^2^ value	—	—	—	—	—	8.734
*P* value	—	—	—	—	—	0.003

## Data Availability

The labeled dataset used to support the findings of this study are available from the corresponding author upon request.
